The article "Nomogram Models Based on the Gene Expression in Prediction of Breast Cancer Bone Metastasis" was published in 2022. Journal: J Healthc Eng.

# Nomogram Models Based on the Gene Expression in Prediction of Breast Cancer Bone Metastasis

**DOI:** 10.1155/2022/8431946

**Published:** 2022-08-22

**Authors:** Teng-di Fan, Di-kai Bei, Song-wei Li

**Affiliations:** Department of Orthopedics, Ningbo Medical Center Lihuili Hospital, Ningbo 315040, Zhejiang, China

## Abstract

**Objective:**

The aim of this study is to design a weighted co-expression network and build gene expression signature-based nomogram (GESBN) models for predicting the likelihood of bone metastasis in breast cancer (BC) patients.

**Methods:**

Dataset GSE124647 was used as a training set, while GSE16446, GSE45255, and GSE14020 were taken as validation sets. In the training cohort, the limma package in *R* was adopted to obtain differentially expressed genes (DEGs) between BC nonbone metastasis and bone metastasis patients, which were used for functional enrichment analysis. After weighted co-expression network analysis (WGCNA), univariate Cox regression and Kaplan–Meier plotter analyses were performed to screen potential prognosis-related genes. Then, GESBN models were constructed and evaluated. The prognostic value of the GESBN models was investigated in the GSE124647 dataset, which was validated in GSE16446 and GSE45255 datasets. Further, the expression levels of genes in the models were explored in the training set, which was validated in GSE14020. Finally, the expression and prognostic value of hub genes in BC were explored.

**Results:**

A total of 1858 DEGs were obtained. The WGCNA result showed that the blue module was most significantly related to bone metastasis and prognosis. After survival analyses, GAJ1, SLC24A3, ITGBL1, and SLC44A1 were subjected to construct a GESBN model for overall survival (OS). While GJA1, IGFBP6, MDFI, TGFBI, ANXA2, and SLC24A3 were subjected to build a GESBN model for progression-free survival (PFS). Kaplan–Meier plotter and receiver operating characteristic analyses presented the reliable prediction ability of the models. Cox regression analysis further revealed that GESBN models were independent prognostic predictors for OS and PFS in BC patients. Besides, GJA1, IGFBP6, ITGBL1, SLC44A1, and TGFBI expressions were significantly different between the two groups in GSE124647 and GSE14020. The hub genes had a significant impact on patient prognosis.

**Conclusion:**

Both the four-gene signature and six-gene signature could accurately predict patient prognosis, which may provide novel treatment insights for BC bone metastasis.

## 1. Introduction

Breast cancer (BC) is one of the most prevalent malignancies and the major cause of cancer-associated deaths of women worldwide [1]. BC is considered to have the highest diagnostic rate in cancer, with more than 1.6 million new cases detected a year, accounting for approximately one-third of all new cancers in women [2]. Substantial improvements in prognosis have been achieved due to better therapeutic approaches over the past 20 years, the overall survival (OS) of BC has increased whereby metastases have become the major cause of death [3]. According to statistics, 627,000 individuals died from BC in 2018, while 684,996 deaths occurred with BC in 2020 [4, 5]. The median OS of patients with metastatic BC ranges from 2 to 3 years, with a 5-year OS rate of 27% [6].

Bone is the common site of metastases, and nearly, 70% of BC patients developed bone metastasis, leading to osteolytic and osteoblastic cancers [7]. Tumor cells secreted factors including the parathyroid hormone in the bone to create an environment conducive to osteolysis instead of the direct destruction of bone [8]. In addition, bone metastasis often contributes to adverse skeletal-related events (SLEs) such as hypercalcemia, nerve root or spinal cord compression, fractures, and pain, which severely affect the quality of life in BC patients [9]. The biggest obstacle to good outcomes in bone metastases is the lack of appropriate therapeutic strategies in the management of tumor-induced SREs [10]. Bone metastases are often challenging because therapies effectively developed against the primary tumor are not satisfactory when used in patients with bone metastases [3]. Currently, magnetic resonance imaging, computed tomography, and X-ray are conventional imaging methods to detect bone metastasis but fail to sense tiny tumor masses and negligible tumor-induced osteolysis [11]. Besides, various metastatic bone lesions which resulted from BC are hard to eradicate by adjuvant localized radiotherapy or surgical intervention [12]. Therefore, it is imperative to identify risk factors and develop predictive models of bone metastases and patient survival to improve the diagnosis and prognosis of bone metastatic BC patients.

High-throughput microarrays have emerged as a promising and efficient tool for studying the complex pathogenesis of human diseases, including cancer [3]. The gene expression also represents an essential role in the prognosis of patients, thus providing clinically relevant information and targeted therapies [13, 14]. Meng et al. constructed a four-long noncoding RNA signature in predicting BC survival based on microarray datasets [15]. Zhao et al. built a gene-expression signature-based nomogram model for the prediction of BC bone metastases, but they did not evaluate the prognostic value of the model [16]. Additionally, a clinical nomogram was constructed to predict bone-only metastasis in patients with early BC [17]. However, the predictive value and independent prognostic significance of the gene expression signature-based nomogram (GESBN) model in bone metastatic BC patients have not been fully elucidated.

On this basis, we constructed a weighted co-expression network using the whole gene expression profile and performed survival analysis to construct predictive nomogram models for bone metastasis that can be used to predict patient OS and progression-free survival (PFS). Besides, the hub genes combined with clinicopathological characteristics were integrated into the nomogram for predicting the occurrence of bone metastases. In addition, we assessed the clinical benefits of the GESBN models and explored their prognostic value in training and validation cohorts. Finally, the expression of the genes in GESBN models and the expression and prognostic value of hub genes were initially explored and validated.

## 2. Materials and Methods

### 2.1. Data Mining from the Gene Expression Omnibus (GEO) Database

The GEO database (https://www.ncbi.nlm.nih.gov/geo/) was used to obtain the BC microarray dataset by setting the following filters: (1) more than 50 samples with BC or bone metastasis information; (2) with survival data; and (3) with expression profiling data. Finally, the GSE124647 dataset was chosen as a training set to identify the DEGs between non-bone metastasis and bone metastasis samples. The platform was Affymetrix Human Genome U133A Array (GPL96). In total, there were 140 samples containing clinical and RNA-seq expression data in the GSE124647 was selected as training cohort. Besides, 107 samples containing OS and RNA-seq expression data in GSE16446, 94 samples containing PFS and RNA-seq expression data in GSE45255 were taken as validation cohorts to verify the prognostic value of GESBN models. Sixty-five samples containing expression data in the GSE14020 dataset were used as validation cohorts to verify the expression levels of key genes. Normalized gene expression was measured as log2-based transformation.

### 2.2. Identification and Functional Enrichment Analysis of DEGs

The *R* package limma was used to screen the DEGs between BC non-bone metastasis and BC bone metastasis groups in the training cohort. |log_2_ FC| > 1 and *P*-value < 0.05 were set as the filtering parameters. Then, Gene Ontology (GO) including biological process (BP), cellular component (CC), and molecular function (MF), and Kyoto Encyclopedia of Genes and Genome (KEGG) were carried out to determine the major biological functions of these DEGs in the database for annotation, visualization, and integrated discovery (DAVID) (https://david.ncifcrf.gov/summary.jsp). *P* < 0.05 was considered statistically significant.

### 2.3. WGCNA

WGCNA is a systemic method that uses gene expression data to build a scale-free network [18]. A weighted co-expression network with the expression profile data of the DEGs was built using the WGCNA package of *R*. Following this, we screened the key module related to BC bone metastasis and prognosis, and then extracted the genes for further analysis.

### 2.4. Nomogram Model Construction and Model Effectiveness Evaluation

In the training cohort, using the “survival” package in *R*, univariate Cox regression analysis was performed to obtain the potential prognostic genes related to OS or PFS. Only genes that had a significant impact on OS or PFS were considered to pass univariate Cox regression analysis screening. In addition, the prognostic value of the significant genes obtained in the univariate Cox regression analysis was evaluated by the Kaplan–Meier plotter analysis. Only genes with statistical significance in OS or PFS analyses were considered to pass the screening. The intersected genes generated in univariate Cox regression and Kaplan–Meier plotter analyses were then entered into the construction of GESBN models in terms of OS and PFS using the “rms” package in *R*. The calibration curves were drawn to measure the performance of the models. The genes which had the greatest contribution were selected as hub genes. Besides, a decision curve analysis (DCA) was performed to assess the clinical net benefit of different models. Further, the hub genes combined with clinicopathological factors were included in the construction of a nomogram for predicting the occurrence of bone metastasis in BC.

After that, the patients were divided into high-risk or low-risk groups using the optimal cut-off value of risk score, which was calculated by the “MaxStat” package in *R*. The Kaplan–Meier plotter analyses were adopted to assess the survival difference between the two groups using “survfit” function of “survival” package in *R*. Moreover, the Cox and ROC analyses were conducted to further evaluate the prognostic value of the GESBN models in training cohort. Subsequently, we verified the prognostic significance of the GESBN models in the validation cohorts. The same method was conducted to compute risk scores like that in the training cohort. The Kaplan–Meier, Cox and ROC analyses were implemented as described earlier. *P* < 0.05 was considered as significantly different. The area under curve (AUC) was used as an indicator of prognostic accuracy.

### 2.5. The Expression Levels of Prognostic Genes in Nomogram Models

The expression levels of key genes between BC nonbone metastasis and BC bone metastasis groups in GSE124647 were first explored using *t* test. Then, GSE14020 as a validation dataset was used to assess the differential expression of the key genes in two groups.

### 2.6. Validation of the Expression and Prognostic Value of the Hub Genes

The protein levels of the hub genes in BC and normal tissues were evaluated using the immunohistochemistry according to the manufacturer's instructions. The Kaplan–Meier plotter (http://kmplot.com/analysis/index.php?p=background) is capable to assess the effect of 54,000 genes on survival in 21 cancer types. We used this database to verify the prognostic significance of the hub genes in BC. Survival curves were generated by the Kaplan–Meier method using the log-rank test. A log-rank *P* value less than 0.05 was statistically significant.

## 3. Results

Figure 1 shows the flowchart of this study.

### 3.1. Identification and Functional Enrichment of DEGs

Taking BC nonbone metastasis samples as a control group, 1858 DEGs in the training set including 992 upregulated and 866 downregulated genes were generated according to the selection criteria. The volcano plot and heat map of the DEGs are presented in Figures 2(a), and 2(b), respectively.

To have a biological understanding of these DEGs, they were subjected to the DAVID database for GO annotation and KEGG pathway enrichment analysis. The top enriched GO terms in BPs were signal transduction, positive regulation of transcription from RNA polymerase II promoter, and immune response, and those in CCs were cytoplasm, cytosol, and extracellular exosome (Figures 3(a) and 3(b)). The major MFs were protein binding, Poly (A) RNA binding, and identical protein binding (Figure 3(c)). In the KEGG pathway enrichment analysis, these genes were mainly involved in the MAPK signaling pathway, proteoglycans in cancer, and focal adhesion (Figure 3(d)). The detailed information for enrichment of GO and KEGG is shown in Table 1.

### 3.2. WGCNA

We incorporated the expression profile of integrated DEGs with clinical traits of the BC samples to construct a gene co-expression network. Clinical characteristics including sample group, PFS time, OS time, OS status, and PFS status were clustered with an expression matrix (Figure 4(a)). Then, we chose the optimal *β* = 6 to ensure that network was scale-free (*β* was a soft-thresholding parameter that could emphasize strong correlations between genes and penalize weak correlations). After choosing the power of 2, the adjacency was transformed into a topological overlap matrix (TOM), which could measure the network connectivity of a gene defined as the sum of its adjacency with all other genes for the network gene ration, and the corresponding dissimilarity (1-TOM) was calculated (Figure 4(b)). Based on TOM, the average linkage hierarchical clustering was conducted to cluster genes by setting the minimum number of genes for each gene network module to 30. To further analyze the module, we calculated the eigen genes of each module and merged the modules by setting a height of 0.25. Finally, 4 modules were acquired (Figures 4(c) and 4(d)). The genes in the grey module could not be incorporated into any other module. Next, Pearson's correlation coefficients of the module eigen gene of each module and the sample characteristics were calculated. The blue module with 76 genes was closely related to bone metastasis and survival status (Figure 4(e)). Thus, the genes in the blue module were chosen for further analysis.

### 3.3. Construction of the GESBN Model

Univariate Cox regression and Kaplan–Meier plotter analyses were carried out on 140 patients in the GSE124647 to evaluate the association of 76 gene expression profiles in the blue module with patient OS and PFS. In univariate Cox regression analysis, significant genes related to OS were SLC44A1, SLC24A3, PDGFC, ITGBL1, and GJA1 (Figure S1A) (all *P* < 0.05). Ten genes including MDFI, IGFBP6, GJA1, ANXA2, SLC24A3, TGFBI, CELA2A, CLEC11 A, PPEF2, and SLC44A1 were notably linked to PFS (Figure S1B) (all *P* < 0.05). However, only four genes related to OS, and six genes related to PFS with statistical differences were extracted in the Kaplan–Meier plotter analysis (Figures S2 and S3) (all *P* < 0.05). Taken together, GAJ1, SLC24A3, ITGBL1, and SLC44A1 were defined as potential prognostic genes for OS. GJA1, IGFBP6, MDFI, TGFBI, ANXA2, and SLC24A3 were potential genes correlated with PFS. These prognostic genes were then subjected to the construction of nomogram models based on OS and PFS (Figures 5(a) and 5(b)). For OS, SLC44A1 had the greatest contribution, which could reach 100 points, while MDFI contributed most to PFS. Therefore, SLC44A1 and MDFI were considered as hub genes. To ensure the accuracy of the GESBN models, the calibration curves for OS and PFS are shown in Figure S4. The DCA results showed that using the nomogram models to predict OS and PFS of patients could increase net benefit compared with other models (Figures 5(c) and 5(d)). For further exploration, we integrate the hub genes and clinicopathological characteristics into the nomogram for predicting the occurrence of bone metastases in BC. As shown in Figure 5(e), progesterone receptor positive (PR+) and early stage increased the bone metastasis risk in BC, indicating that bone metastases more frequently occurred in less aggressive and earlier stage BC patients.

### 3.4. Evaluation of the GESBN Models

The GESBN score was calculated for each patient in the training set. Patients were ranked based on their risk scores and assigned into two groups as high-risk and low-risk of bone metastases. Kaplan–Meier survival analysis in the training cohort showed that the OS rate of patients in the high-risk group was low, and the difference between the two groups was statistically significant (Figure 6(a)) (*P* < 0.001). Similarly, an unfavorable PFS was observed in the high-risk group patients (Figure 6(b)) (*P* < 0.001), suggesting that two GESBN models could predict survival well. Further, the time-dependent ROC curves were drawn using the pROC package in *R*. In terms of OS, the AUCs of the 3- and 5-year survival rates were 0.62, and 0.72, respectively (Figure 6(c)). For PFS, the AUCs of the 3- and 5-year survival rates were 0.88, and 0.94, respectively (Figure 6(d)), indicating that GESBN models had a good predictive ability. We further evaluate the efficacy of the GESBN models in predicting OS and PFS in the validation cohorts. Consistent with the previous results, patients in the high-risk group had significantly shorter OS and PFS time than that in the low-risk group (Figures 7(a) and 7(b)). The time-dependent ROC analyses also showed that the GESBN models had favorable performance in predicting OS and PFS (Figures 7(c) and 7(d)).

Moreover, to investigatealyses were carried out in the training and validation cohorts. In the training cohort, univariate analysis exhibited that progesterone receptor (PR) status and four-gene risk score were significantly related to OS, while PR status, prior endocrine sensitivity, and six-gene risk score had close relationship with PFS (all *P* < 0.05). In the multivariate analysis, GESBN models were independent predictors for OS (HR = 2.289, 95% CI: 1.253–4.180, *P* < 0.01) and PFS (HR = 2.624, 95% CI: 1.757–3.919, *P* < 0.001) (Table 2). Consistently, the GESBN models displayed pronounced capability in predicting OS and PFS in the validation cohorts (all *P* < 0.05) (Table 3). These results suggested that the GESBN models were independent variables.

Following this, ROC analyses were conducted to evaluate how the GESBN models behaved in predicting prognosis. The results showed that the AUC of the four-gene risk score model performed on OS in the training cohort was 0.691, which was better than that of PR status, prior endocrine sensitivity, and stage (0.524, 0.540, and 0.503, respectively) (Figure 8(a)). In the prediction model of PFS predicted in the training cohort, the six-gene risk score also exhibited a powerful ability with AUC = 0.758, which was superior to other variables (Figure 8(b)). The same results were observed in the validation cohorts (Figures 8(c) and 8(d)).

### 3.5. The Expression Levels of Genes in GESBN Models

Due to the predictive ability of GESBN models for both OS and PFS, we explored the expression levels of these key genes. In the training dataset of GSE124647, the expression levels of all the prognosis-related genes were significantly different between control and bone-metastasis groups (Figure 9(a)) (all *P* < 0.05). In the validation dataset of GSE14020, GJA1, IGFBP6, ITGBL1, SLC44A1, and TGFBI expressions in the bone-metastasis group were different from those in the control group. The differences were statistically significant (Figure 9(b)) (*P* < 0.05).

### 3.6. Validation of the Expression and Prognostic Value of Hub Genes

Based on the GESBN result, SLC44A1 and MDFI were the hub genes. The immunohistochemistry images showed that the protein levels of SLC44A1 were higher in BC tissue than that in normal breast tissue (Figures 10(a) and 10(b)). Similarly, an elevated MDFI expression was observed in the BC tissue compared with the normal breast tissue (Figures 10(c) and 10(d)). The Kaplan–Meier plotter was performed to verify the effect of SLC44A1 and MDFI on OS, PFS, and DMFS in BC. Patients in the high SLC44A1 expression group tended to have favorable OS, PFS, and DMFS (Figures 11(a)–11(c)) (*P* < 0.05). Although the MDFI expression was not significantly linked to OS and DMFS of the BC patients (Figures 11(d) and 11(f)) (*P* > 0.05), its high expression predicted worse PFS (Figure 11(e)) (*P* < 0.01). These results indicated that SLC44A1 and MDFI might be potential biomarkers for BC.

## 4. Discussion

BC is a heterogenous tumor driven by various molecular progression pathways [19]. Analyses of BC progression showed that bone is the first metastatic site of this disease possibly due to the favorable chemokine milieu or microenvironment in the bone, as well as the intrinsic molecular characteristics of cancer cells [17, 20]. Although these hypotheses are promising, biological information and anatomical characteristics are still the basis for clinicians to determine prognosis; however, the predictors of bone metastasis remain uncertain clinically [17, 21]. Some gene signature-based prognostic prediction models for BC patients have been reported via repurposing and analysis of microarray data [22, 23]. These models were built for predicting OS for BC patients but lack the prediction of bone metastasis. By using GEO accession number GSE124647, we obtained 1858 DEGs between BC nonbone metastasis and bone metastasis groups. After screening the prognosis-related genes, we constructed a four-gene expression signature-based nomogram model and a six-gene expression signature-based nomogram model.

We first conducted a differential analysis of the GSE124647 dataset in relation to BC bone metastasis and employed functional enrichment analysis to these DEGs, which were found to be mainly related to signal transduction, and positive regulation of transcription in terms of BP. CCs were mainly enriched in cytoplasm and cytosol. MFs were mainly protein binding, and Poly (A) RNA binding. The potential pathways that they were involved in were MAPK signaling pathway and proteoglycans in cancer. Based on WGCNA, 76 genes in the blue module were initially selected for the following prognostic analysis. After univariate Cox regression and Kaplan–Meier plotter analyses, OS nomogram including GJA1, SLC24A3, ITGBL1, and SLC44A1, and PFS nomogram including GJA1, IGFBP6, MDFI, TGFBI, ANXA2, and SLC24A3 were constructed. Among them, SLC44A1 and MDFI were considered as hub genes. Since BC is a molecularly heterogenous disease which similar tumors form various clinical outcomes and metastases patterns [24]. It has been demonstrated that BC luminal subtype and patients at low-grade are more prone to develop metastases [16]. Considering the organ-specific tendency of metastasis regarding molecular subtypes, we constructed a model containing hub genes and clinicopathological characteristics for predicting the occurrence of BC bone metastases. Consistently, we found that PR+ and early stage increased the bone metastatic risk of BC patients. Thus, the authors speculated that despite the development of bone metastases, the patient's tumor is still of low malignancy and the clinical outcome might be improved if the bone lesions are well controlled. Then, Kaplan–Meier plotter, Cox and ROC analyses confirmed the reliable and superior prognostic ability of GESBN models. AUC can be used to assess the accuracy and predictive capacity of biomarkers in diagnostic tests [25].

After confirming the predictive value of nomograms, we validated the expression and prognostic significance of hub genes in the models. Expectedly, SLC44A1 and MDFI protein levels were higher in BC tissues than those in normal breast tissues. We found that the high SLC44A1 expression was significantly related to favorable OS, PFS, and DMFS. However, patients in the high MDFI group predicted worse PFS. The solute carrier (SLC) superfamily contains various membrane-bound transporters which are required to transport a wide variety of substrates over biological membranes, and the dysregulated expression of these transporters may be related to cancer metastasis. SLCO1B1 was found to be highly expressed in colon cancer, and its expression level was significantly associated with the degree of differentiation in this type of cancer [26]. SLCO1B3 overexpression may be linked to hormone-dependent growth mechanisms, and the expression of this transporter could serve as a valid prognostic factor for BC [27]. As a member of the SLC superfamily, SLC44A1 is a mitochondrial protein mediating choline transport and is preferentially expressed in neurons and oligodendrocytes [28]. Besides, high activity of the SLC44A1 promoter has been proved to participate in the occurrence of papillary glioneuronal tumors [29]. Our study revealed an important finding that high SLCO4A1 expression contributed to the favorable clinical outcome for BC metastasis patients. MDFI is a transcription factor that negatively regulates myogenic family proteins [30]. A previous study has demonstrated that the loss of MDFI was related to human BC and myeloid neoplasm via negative regulation of the Wnt pathway [31]. In this study, high MDFI expression led to poor PFS for patients with metastatic BC.

## 5. Conclusions

Based on the construction of a weighted co-expression network for DEGs between BC nonbone metastasis and bone metastasis, we screened the key module and related genes to investigate a prognostic nomogram model for bone metastatic BC. The study provided some potent biomarkers of BC bone metastasis and enabled the prediction of patient survival. We also found that SLC44A1 and MDFI were the hub genes in BC bone metastasis, which might be the therapeutic targets for this disease.

## Figures and Tables

**Figure 1:** Flowchart showing the analysis process.

**Figure 2:** Differentially expressed genes between breast cancer nonbone metastasis and bone metastasis patients from the GSE124647 dataset. (a) Volcano plot of the 992 upregulated (red triangle) genes and 866 downregulated (green triangle) genes. (b) Heat map of the top 50 significant differentially expressed genes.

**Figure 3:** Functional enrichment analysis of differentially expressed genes. (a) Biological process. (b) Cellular component. (c) Molecular function. (d) KEGG pathway.

**Figure 4:** Weighted co-expression network analysis. (a) Dendrogram of sample clustering and heatmap of clinical traits of all breast cancer samples in a dataset of GSE124647. (b) The optimal *β* value result graph. (c) Module eigen gene dendrogram. The horizontal axis represents a color block, and each of the different color blocks represents a different module, and the vertical axis represents the height of the dendrogram based on the expression value. (d) Clustering of module eigen genes. (e) The correlation between gene modules and sample characteristics.

**Figure 5:** Gene expression signature-based nomogram models and decision curve analysis (DCA). (a) The four-gene-based nomogram model based on overall survival (OS). (b) The six-gene-based nomogram model based on progression-free survival (PFS). (c) DCA for the nomogram model based on OS. Model 1: GJA1; model 2: GJA1 + SLC24A3; model 3: nomogram. (d) DCA for the nomogram model based on PFS. Model 1: IGFBP6 + GJA1; model 2: IGFBP6 + GJA1 + TGFBI + MDFI; model 3: nomogram. (e) Construction of nomogram model for predicting bone metastasis. PR status, progesterone receptor status, 0: negative, 1: positive; PES, prior endocrine sensitivity.

**Figure 6:** Prognostic evaluation of gene expression signature-based nomogram models in GSE124647. Kaplan–Meier plotter. (a) Overall survival curve and (b) progression-free survival curve between high-risk and low-risk bone metastatic patients. (c) Receiver operating characteristic (ROC) analysis of the four-gene signature. (d) ROC analysis of the six-gene signature. Abbreviations: L, low; H, high; HR, hazard ratio.

**Figure 7:** Prognostic evaluation of gene expression signature-based nomogram models in validation cohorts. (a) Kaplan–Meier plotter overall survival curve in GSE16446. (b) Kaplan–Meier plotter progression-free survival curve in GSE45255. (c) Receiver operating characteristic (ROC) analysis of the four-gene signature in GSE16446. (d) ROC analysis of the six-gene signature in GSE45255. Abbreviations: L, low; H, high; HR, hazard ratio.

**Figure 8:** Receiver operating characteristic (ROC) analysis of the gene expression signature-based nomogram models in the training and validation cohorts. (a) ROC analysis of the predictive value of PR status, PES, stage, and four-gene risk score in the training cohort based on OS. (b) ROC analysis of the predictive value of PR status, PES, stage, and six-gene risk score in the training cohort based on PFS. (c) ROC analysis of the predictive value of PR status, PES, stage, and four-gene risk score in the GSE16446 as validation cohort based on OS. (d) ROC analysis of the predictive value of PR status, PES, stage, and six-gene risk score in the GSE16446 as validation cohort based on PFS. PR status, progesterone receptor status; PES, prior endocrine sensitivity; OS, overall survival; PFS, progression-free survival.

**Figure 9:** Expression levels of genes in gene expression signature-based nomograms. (a) GSE124647. (b) GSE14020.

**Figure 10:** The protein expression levels of SLCC4A1 and MDFI. The protein expression levels of SLC44A1 in (a) breast cancer tissue and (b) normal breast tissue. The protein expression levels of MDFI in (c) breast cancer tissue and (d) normal breast tissue.

**Figure 11:** Prognostic value of the hub genes in breast cancer. The effect of SLC44A1 on (a) overall survival, (b) progression-free survival, and (c) distant metastasis-free survival in breast cancer patients. The effect of MDFI on (d) overall survival, (e) progression-free survival, and (f) distant metastasis-free survival. Abbreviations: HR, hazard ratio.

**Table 1:** GO annotation and KEGG pathway analyses of differentially expressed genes.

Category	Term	Count	*P*-value
GO annotation KEGG pathway	Signal transduction	170	9.70 *E* − 07
	Positive regulation of transcription from RNA polymerase II promoter	147	1.59 *E* − 06
	Immune response	84	2.93 *E* − 09
	Inflammatory response	81	2.00 *E* − 10
	Response to lipopolysaccharide	44	4.43 *E* − 09
	Extracellular exosome	421	5.95 *E* − 22
	Cytosol	442	1.98 *E* − 13
	Extracellular space	209	6.48 *E* − 12
	Cytoplasm	626	3.36 *E* − 10
	Membrane	294	6.25 *E* − 09
	Protein binding	1047	2.72 *E* − 14
	Poly(A) RNA binding	166	1.02 *E* − 06
	IgG binding	8	2.63 *E* − 05
	Double-stranded RNA binding	18	9.01 *E* − 05
	Identical protein binding	109	1.37 *E* − 04

KEGG pathway	Platelet activation	35	1.01 *E* − 05
	Phagosome	33	1.06 *E* − 03
	Proteoglycans in cancer	39	3.52 *E* − 03
	Lysosome	26	5.54 *E* − 03
	MAPK signaling pathway	46	5.81 *E* − 03
	Focal adhesion	39	5.88 *E* − 03
	Drug metabolism - other enzymes	13	7.84 *E* − 03
	Regulation of actin cytoskeleton	39	8.11 *E* − 03
	Leukocyte transendothelial migration	24	0.011
	Chemical carcinogenesis	18	0.015

Abbreviations. GO, Gene Ontology; KEGG, Kyoto Encyclopedia of Genes and Genomes.

**Table 2:** Cox regression analysis of the GESBN models and clinical variables in the training cohort.

Overall survival				
Variables	*Univariate analysis*		*Multivariate analysis*	
	HR (95% CI)	*P* value	HR (95% CI)	*P* value
PR status	0.552 (0.363–0.838)	0.005	0.660 (0.398–1.094)	0.107
PES	0.644 (0.403–1.029)	0.066	0.649 (0.405–1.040)	0.073
Stage	1.006 (0.656–1.543)	0.979	1.214 (0.673–2.192)	0.519
Risk score	2.719 (1.663–4.447)	<0.001	2.289 (1.253–4.180)	0.007

*Progression-free survival*				
PR status	0.598 (0.420–0.853)	0.004	0.807 (0.531–1.228)	0.317
PES	0.600 (0.395–0.912)	0.017	0.657 (0.424–1.016)	0.059
Stage	0.750 (0.517–1.088)	0.129	1.006 (0.604–1.674)	0.983
Risk score	2.710 (1.920–3.824)	<0.001	2.624 (1.757–3.919)	<0.001

abrAbbreviations: GESBN, gene expression signature-based nomogram; HR, hazard ratio; 95% CI, 95% confidence interval; PR status, progesterone receptor status; PES, prior endocrine sensitivity.

**Table 3:** Cox regression analysis of the GESBN models and clinical variables in the validation cohorts.

Overall survival				
Variables	*Univariate analysis*		*Multivariate analysis*	
	HR (95% CI)	*P* value	HR (95% CI)	*P* value
N stage	0.856 (0.388–1.887)	0.700	0.761 (0.343–1.687)	0.501
Grade	1.210 (0.364–4.019)	0.756	1.198 (0.337–4.265)	0.780
T stage	1.696 (0.980–2.930)	0.059	1.407 (0.827–2.393)	0.208
Risk score	2.719 (1.300–5.686)	0.008	2.442 (1.130–5.227)	0.023

*Progression-free survival*				
Grade	1.635 (0.792–3.374)	0.184	1.323 (0.535–3.272)	0.545
Age	1.022 (0.987–1.058)	0.227	1.037 (0.996–1.080)	0.074
PR status	0.333 (0.133–0.835)	0.019	0.572 (0.194–1.686)	0.311
Risk score	2.714 (1.582–4.655)	<0.001	2.773 (1.469–5.235)	0.002

abrAbbreviations. GESBN, gene expression signature-based nomogram; HR, hazard ratio; 95% CI, 95% confidence interval; PR status, progesterone receptor status.

## Data Availability

The dataset used and/or analyzed during the current study are available from the corresponding author on reasonable request.

## Supplementary Materials

Supplementary Materials Figure S1. Forest plot of univariate Cox regression analyses of prognosis. (A) Significant genes related to overall survival. (B) Significant genes related to progression-free survival. Figure S2. Prognostic genes related to overall survival by Kaplan-Meier plotter. Abbreviations: (L) Low; (H) High; HR, Hazard ratio. Figure S3. Prognostic genes related to progression-free survival by Kaplan-Meier plotter. Abbreviations: (L) Low; (H) High; HR, Hazard ratio. Figure S4. Calibration curves of gene expression signature-based nomogram models. (A) Calibration curve for predicting patient overall survival. (B) Calibration curve for predicting patient progression-free survival.
